# Molecular Typing Based on Oxidative Stress Genes and Establishment of Prognostic Characteristics of 7 Genes in Lung Adenocarcinoma

**DOI:** 10.1155/2022/9683819

**Published:** 2022-09-12

**Authors:** Jing Tu, Min Tang, Guoqing Li, Liang Chen, Yong Huang

**Affiliations:** ^1^Department of Pulmonary and Critical Care Medicine, Chongqing General Hospital, No. 118, Xingguang Avenue, Liangjiang New Area, Chongqing 401147, China; ^2^Department of Oncology, Chongqing General Hospital, No. 118, Xingguang Avenue, Liangjiang New Area, Chongqing 401147, China; ^3^Intensive Care Unit, Chongqing General Hospital, No. 118, Xingguang Avenue, Liangjiang New Area, Chongqing 401147, China

## Abstract

Oxidative stress could maintain different biological processes in human cancer. However, the effect of oxidative stress on lung adenocarcinoma (LUAD) should be studied. This study analyzed the expression and clinical importance of oxidative stress in LUAD in detail. The Cancer Genome Atlas (TCGA) and Gene Expression Omnibus (GEO) were employed for obtaining LUAD expression profiles. Based on oxidative stress-related genes, molecular subtypes substantially correlated with the LUAD prognosis were discovered with ConsensusClusterPlus. Differentially expressed genes (DEGs) among subtypes were found using the Limma software package. Least absolute shrinkage and selection operator- (Lasso-) Cox analysis was employed to create the polygenic risk model. RiskScore and clinically relevant features were used to create nomograms. By utilizing oxidative stress-related genes and reliable clustering, stable molecular subtypes were first discovered. The prognosis, clinical characteristics, route characteristics, and immunological characteristics of these three molecular subtypes were all different. Subsequently, by using differential expression genes among molecular subtypes and Lasso, 7 main genes linked with the oxidative stress phenotype were discovered. A prognostic risk model was also built on the basis of major genes associated with the oxidative stress phenotype. The model demonstrated a high level of resilience and was unaffected by clinical-pathological features. It played a stable predictive role in independent datasets. Ultimately, to improve the prognosis model and survival prediction, RiskScore (RS) was combined with clinicopathological variables, and a decision tree model was used. The model exhibited a high prediction accuracy as well as the ability to predict survival. This research found that oxidative stress-related genes have a major involvement in the onset and progression of LUAD and that they may influence LUAD susceptibility to immunotherapy and standard chemotherapy. Furthermore, the identified risk models for 7 genes linked with oxidative stress exhibited could assist clinical treatment decisions and prognosis prediction. The classifier could be used as a molecular diagnostic tool for assessing LUAD patients' prognosis risk.

## 1. Introduction

Lung cancer is among the most widely known fatal malignancy with the highest occurrence and death rate in people of both genders around the globe [1]. According to pathological classification, lung cancer can be categorized as small-cell lung adenocarcinoma and non-small-cell lung cancer (NSCLC), among which the latter accounts for about 2/3 cases [2]. NSCLC can be divided into three types, including lung adenocarcinoma, squamous cell lung cancer, and non-small-cell lung cancer, of which lung adenocarcinoma (LUAD) accounts for about 40% of cases [3]. LUAD is classified as the most widely known histological subtype of cancer, with annual new cases of approximately 2.09 million and 1.76 million deaths [4]. Although progress has been made in the methods to treat LUAD, due to patient heterogeneity, the quality of life of patients has not improved yet, and the 5-year overall survival rate (OS) of LUAD patients remains at 16% [5]. Consequently, specific prognostic strategies for LUAD patients are urgently needed to discover novel therapeutic targets and improve patient survival rates.

Tobacco smoke comprises a complex variety of chemical compounds, for instance, reactive oxygen species (ROS) and reactive nitrogen species (RNS), which can degrade macromolecular targets like lipids, proteins, and nucleic acids [6]. Growing evidence suggests that smoking-induced ROS and the oxidative stress that results play an increasingly essential role in inflammation and cancer. Approximately 90% of lung cancer cases are directly linked to smoking [7]. Oxidative stress means the overproduction of molecules that are highly active in the body, including ROS and RNS, when the body needs to remove aging cells or when it is exposed to a variety of harmful stimuli, and the oxidation degree exceeds the oxides' removal, resulting in tissue deterioration and an imbalance between the oxidation system and the antioxidant system [1]. Oxidative stress appears to be greatly involved in the pathogenesis of a variety of ailments, e.g., inflammatory diseases, cancer, and immune-mediated diseases, according to numerous studies [8]. The dynamic interaction between diverse cells in the tumor microenvironment (TME) has been shown in a multitude of studies to affect the redox status of each cell group [9]. A fundamental regulator of carcinogenesis is the tumor microenvironment, which consists of endothelial cells, fibroblasts, tumor cells, macrophages, immune cells, and an extracellular matrix. It has a substantial impact on the occurrence, development, and progression of LUAD and the responsiveness to a variety of treatment options [10]. ROS has been increasingly considered having a complicated and diversified impact on the tumor microenvironment recently. Tumor redox has the ability to target and enhance the oxidative stress within the tumor, resulting in tumor necrosis.

Growing research indicates that cancer immunotherapy can alter tumor oxidation-reduction, resulting in aggravated tumor oxidative stress and ROS-dependent tumor rejection [11]. Hence, we hypothesized that oxidative stress affects the progression of LUAD and investigated whether there is significant difference in oxidative stress-related subtypes of LUAD, thus providing a theoretical basis for optimizing immunotherapy or developing new treatment plans.

The genes of the oxidative stress pathway were employed in this investigation to define stable molecular subtypes through reliable clustering, and clinical, pathway, and immunological characteristics were compared between subtypes. Then, with the help of the least absolute shrinkage and selection operator (Lasso), genes associated with the oxidative stress phenotype were discovered. A risk model and a clinical prognosis model were also developed, which might be utilized to help with lung adenocarcinoma patients' prognosis and individualized treatment.

## 2. Materials and Methods

### 2.1. Data Collection and Processing

The cancer genome map was utilized to retrieve LUAD mutation and copy number variation data from The Cancer Genome Atlas (TCGA) database. TCGA GDC API was employed for downloading the RNA sequencing (RNA-seq) data from TCGA-LUAD. The Gene Expression Omnibus (GEO) database was employed to get the expression data for GSE31210 [12] and GSE50081 [13]. The training set in this work was TCGA-LUAD, while the independent verification sets were GSE31210 and GSE50081.

### 2.2. Data Preprocessing

The following steps were used to preprocess the RNA-seq data from TCGA-LUAD dataset: (1) samples with no clinical follow-up data were deleted, (2) samples with no survival time were excluded, (3) samples with no status were eliminated, (4) Ensembl was changed to a gene symbol, and (5) an expression containing several gene symbols was assigned the middle value. The following steps were followed to preprocess the GEO data: for the GEO dataset, the annotation data for the relevant chip platform was obtained, the probe was mapped to the gene using the annotation information, and probes that matched multiple genes were eliminated. When numerous probes matched the same gene, the median was considered the gene expression value.

### 2.3. Molecular Subtypes of Genes Related to Oxidative Stress

Our oxidative stress genes were from the Molecular Signatures Database's (MSigDB) “GOBP RESPONSE TO OXIDATIVE STRESS” oxidative stress pathway [14]. ConsensusClusterPlus was employed for creating a consistency matrix on the basis of gene expression profiles, and the samples were clustered and typed [15]. The expression data of genes related to oxidative stress was employed to determine sample molecular subtypes. The distance was measured using the “km” algorithm and “1-Spearman correlation” using 500 bootstraps. 80% of the training set patients were added in each bootstrap process. The number of clusters was set to 2 to 10, and the molecular subtypes of the samples were established by computing the consistency matrix and the consistency cumulative distribution function.

### 2.4. Construction of the Risk Model

Initially, the oxidative stress genes that were expressed differentially among the subtypes were discovered with the help of molecular subtypes identified previously. Afterward, we chose the genes that were expressed differentially (|log2fold change (FC)| > 1 and *p* < 0.05) with a high prognosis. Furthermore, Lasso regression was done to lower the number of genes, and the prognostic genes linked with the oxidative stress phenotype were retrieved. Finally, we made the risk model. For every patient, the RiskScore (RS) was measured with the help of the formula stated: RS = *Σβ* *i* × Exp *i*), where “*i*” refers to the expression degree of genes linked with the prognosis of the oxidative stress phenotype and “*β*” is the Cox regression coefficient of the related gene. As per the threshold value “0,” patients were sorted into high-RS and low-RS groups. The Kaplan-Meier method was employed for drawing the survival curve for prognosis analysis, and the log-rank test was performed for finding the importance of the variation.

### 2.5. Gene Set Enrichment Analysis (GSEA)

For analyzing the pathways of various biological activities in distinct molecular subtypes, we utilized the “GSEA.” In this study, all candidate gene sets from the Hallmark database [14] were utilized for GSEA. The oxidative stress pathway was provided by the “WP_FERROPTOSIS” in the MSigDB. The autophagy pathway was taken from “GOBP_REGULATION_OF_AUTOPHAGY” in the MSigDB. Gene sets linked with inflammatory features and angiogenesis were obtained from the previous literature [16, 17].

### 2.6. Calculation of Invasion Abundance of TME Cells

In lung adenocarcinoma, the CIBERSORT algorithm (https://cibersort.stanford.edu/) was employed to quantify the relative number of 22 immune cells [18]. Simultaneously, the ESTIMATE software was used to measure the proportion of immune cells, and the Wilcoxon test was employed to evaluate the degree of immune cell infiltration in the high-RS and low-RS groups [19].

### 2.7. Prediction of Responsiveness to Immunotherapy

The impact of IMS on the prediction of clinical responsiveness of immune checkpoint inhibitors (ICIs) was tested using the tumor immune dysfunction and exclusion (TIDE) algorithm. The TIDE algorithm is a mathematical approach that employs gene expression profiles to estimate immune checkpoint blockade response [20]. The TIDE algorithm evaluated three cell types that limited tumor T cell infiltration, including the M2 subtype of tumor-associated fibroblasts (CAFs), myeloid-derived suppressor cells (MDSCs), and tumor-associated macrophages (TAMs), as well as two distinct tumor immune escape mechanisms, such as T cell exclusion score of immunosuppressive factors on cytotoxic T lymphocytes (CTLs) and T cell dysfunction score of tumor infiltration.

### 2.8. Construction and Verification of Nomograph

The nomogram can display the risk model's outcomes visually and effectively, making it easier to predict them. The nomograph employs line length to depict the impact of various variables and variable values on the outcomes. A nomogram model [21] was created based on the outcome of the univariate and multivariate analyses.

### 2.9. Statistical Analysis

R (https://www.r-project.org/, version 3.6.3) helped in all statistical analyses and data visualization. All estimated *p* values were double-tailed, with a significance level of *p* < 0.05.

## 3. Results

### 3.1. Three Oxidative Stress Subtypes in LUAD Based on Consensus Clustering of Oxidative Stress-Related Genes

The flow chart of the whole study is shown in Figure S1. Univariate Cox regression analysis indicated that 102 oxidative stress genes were linked with the lung adenocarcinoma prognosis in TCGA-LUAD dataset (Supplementary Table S1, *p* < 0.05). As per the expression degree of these 102 oxidative stress genes, patients were categorized following consistent clustering of gene expression profiles, and the optimal number of clusters was found using the cumulative distribution function (CDF). The CDF delta area curve revealed that upon selection of the cluster as 3, comparatively stable clustering outcomes were received (Figures 1(a) and 1(b)). Consequently, LUAD patients were sorted into three oxidative stress-related subtypes: C1, C2, and C3 (Figure 1(c)). In TCGA-LUAD cohort, major variations were observed in the prognosis of the three clusters linked with oxidative stress (*p* < 0.05, Figure 1(d)). Generally, C3 had a good prognosis, while the prognosis of C1 was poor. We also carried out a comparison of the variations in the expression of 102 oxidative stress genes in various molecular subtypes that we defined (Figure 1(e)); it was discovered that the “risk” gene was substantially expressed in subtype C1, while the “protective” gene was highly expressed in the C3 subtype. Additionally, we measured the “oxidative stress single-sample gene set enrichment analysis (ssGSEA) scores” of each patient suffering from lung adenocarcinoma in TCGA-LUAD cohort. The outcomes highlighted that C2 and C3 subtypes had greater “oxidative stress ssGSEA scores” (Figure 1(f)).

### 3.2. Link between Oxidative Stress Subtypes and Clinical Properties

The link between the three oxidative stress subtypes and clinical-pathological variables was then investigated, and proportional distribution maps of various clinical features were produced. T stage (Figure 2(a)), N stage (Figure 2(b)), stage (Figure 2(d)), age (Figure 2(e)), gender (Figure 2(f)), and status (Figure 2(g)) exhibited significant differences in TCGA-LUAD cohort, but M stage showed no significant differences (Figure 2(c)). The findings revealed that the C1 subtype had a larger proportion of nonearly clinical stages than the C2 and C3 subtypes (Figures 2(a)–2(d)). Moreover, C1 subtypes had the majority of male patients (Figure 2(f)) with a relatively higher death rate (Figure 2(g)), which was consistent with the poor prognosis in this group.

### 3.3. Comparison of Somatic Variation of the Three Oxidative Stress Subtypes

In TCGA-LUAD cohort, the variations in genomic alterations among these three molecular subtypes were also investigated. The earlier pan cancer study [22] provided information about molecular properties of TCGA-LUAD. Subtype C1 had higher homologous recombination defects, fraction altered, aneuploidy score, number of segments, and tumor mutation burden, as per the findings (Figure 3(a)). Additionally, we performed a comparison between the relationship of the five known immune molecular subtypes and the three types of molecular subtypes that we discovered, and it was observed that C3 subtypes of the immune molecular subtypes defined by us occupied more of them (Figure 3(b)), and the best prognosis was noticed in the C3 subtypes of the existing immune subtypes among the five types of subtypes, which was similar to the outcomes of our definition of subtypes. Furthermore, a comparison was carried out between the differences in gene mutations in various molecular subtypes. The top 20 genes with significant mutations were highlighted. We discovered that most mutations were present in MUC16, KEAP1, and CDH10, accounting for 52.7%, 23.9%, and 22.6%, respectively, and the mutation type was mainly missense mutations (Figure 3(c)). Those data indicated that the C3 subtype with better survival time had lower gene mutation.

### 3.4. Immune Characteristics of the Three Oxidative Stress Subtypes and Differences in Immunotherapy/Chemotherapy

The immunological features of the three oxidative stress subtypes were studied to assess immune heterogeneity among the three oxidative stress subtypes. CIBERSORT was employed for measuring the relative abundance of 22 immune cells, and a comparison between the three subtypes was done (Figure 4(a)). Major variations in TCGA-LUAD cohort were displayed by the following: (1) plasma cells, (2) B cells memory, (3) T cells CD8, (4) activated memory CD4 T cells, (5) resting memory CD4 T cells, (6) helper follicular T cells, (7) activated NK cells, (8) resting NK cells, (9) monocytes, (10) M0 and M1 macrophages, (11) activated dendritic cells, (12) resting dendritic cells and activated mast cells, and (13) resting mast cells. The immune cell infiltration was also analyzed simultaneously using ESTIMATE (Figure 4(b)). It could be seen that the “immune score” of subtypes C2 and C3 was considerably higher in comparison with that of subtype C1, with greater immune cell infiltration.

Then, we studied if molecular subgroups in TCGA cohort had varying responses to immunotherapy. The expression of immunological checkpoints was evaluated between subtypes, and 44 immune checkpoint genes were identified to be differently expressed (Figure 4(c)). The TIDE score of the C3 subtype in TCGA cohort was found to be lower in comparison with that of the other two subtypes, indicating that immunotherapy was more beneficial to it (Figure 4(d)). In addition, we looked at how distinct molecular subtypes in TCGA cohort responded to the standard chemotherapy medications Docetaxel, Vinorelbine, Paclitaxel, and Cisplatin and discovered that the IC50 of the four chemotherapy medicines varied significantly between the three subtypes. C1 was also more responsive to Docetaxel, Vinorelbine, and Cisplatin than other kinds (Figure 4(e)). Those findings showed that patients in the C3 subtype presented high immune infiltration status.

### 3.5. Pathway Characteristics among the Three Molecular Subtypes

The variations in activated pathways between molecular subtypes were investigated further. The findings indicate that 33 pathways were considerably enriched in TCGA cohort's C1 subtype. Activated pathways included (1) HALLMARK DNA REPAIR, (2) HALLMARK E2F TARGETS, (3) HALLMARK MYC TARGETS V2, (4) HALLMARK MYC TARGETS V1, etc. (Figure 5(a)). When comparing the different pathways between different C2 subtypes and other subtypes, it was discovered that the pathways involved in tumor development in patients with C2 subtypes were activated as a whole; these included (1) HALLMARK EPITHELIAL MESENCHYMAL TRANSITION, (2) HALLMARK TGF BETA SIGNALING, (3) HALLMARK NOTCH SIGNALING, etc. (Figure 5(a)). Moreover, it was discovered that the pathways related to the cell cycle in the C3 subtype were inhibited as a whole (Figure 5(a)).

Furthermore, the three molecular subtypes' inflammatory actions were investigated. Except for “STAT1,” the ssGSEA scores of the C2 and C3 subtypes in the other six metagenes were higher than those of the C1 subtype (Figure 5(b)). The three molecular subtypes also had substantial variation in the ssGSEA scores of ferroptosis, autophagy, and angiogenesis. The C1 subtype exhibited the highest rate of iron mortality but the lowest rates of autophagy and angiogenesis (Figures 5(c)–5(e)).

### 3.6. Identification of Key Genes of the Oxidative Stress Phenotype

747 genes were chosen after identifying the differently expressed genes among molecular subtypes (false discovery rate (FDR) < 0.05 and |log2FC| > 1), and the differentially expressed genes among subtypes were examined using univariate Cox regression. A total of 337 genes (*p* < 0.01) were found to have a significant impact on the prognosis, including 202 “risk” and 135 “protective” genes (Figure 6(a)). These genes are enriched in many pathways, such as cell cycle-related pathways (Figure S2). Lasso cox regression was used once more.  Figure 6(b) depicts the changing track of each independent variable. It can be seen that lambda increased along with the number of independent variable coefficients that tended to be 0. The model was best when lambda = 0.0554, as illustrated in Figure 6(c). As a result, with lambda = 0.0554, 20 genes were chosen as target genes in the next stage. In the ideal model, stepwise Akaike information criterion (stepAIC) in the mass package lowered the genes from 13 to 6 and estimated the risk value of each gene. Finally, seven genes (MELTF, PTPRH, LOXL2, RHOV, CPS1, IRX5, and MS4A1) were identified as oxidative stress-related genes that influenced the prognosis (MELTF, PTPRH, LOXL2, RHOV, CPS1, IRX5, and MS4A1) (Figure 6(d)).

### 3.7. Generation and Validation of the RS Model Based on 7 Genes Related to Oxidative Stress

The expression and coefficients of seven genes linked with oxidative stress were employed for creating a prognostic model linked with oxidative stress and for measuring the risk value of LUAD samples and ranking them. Based on the dividing point, those with RS greater than 0 were categorized as high risk, and those with RS less than or equal to 0 were categorized as low risk. Therefore, we sorted 253 samples into the low-RS group and 247 samples into the high-RS group. The risk map of TCGA-LUAD revealed the expression, survival status, and risk value distribution of 7 genes linked with oxidative stress in each LUAD patient (Figure 7(a)), which indicated that samples with high RS had a poor prognosis. The prognosis categorization of RS was then subjected to ROC analysis. The model exhibited a high area under the AUC line (1-year AUC = 0.74, 3-year AUC = 0.74, and 5-year AUC = 0.69), indicating that it had a good classification efficiency of prognosis prediction in one, three, and five years (Figure 7(b)). The prognosis of the high-RS group was poorer (*p* < 0.0001, Figure 7(c)), and a major variation was noted in the survival time of the high-RS and low-RS groups. Validation analysis results were performed in two more independent lung adenocarcinoma cohorts to corroborate the robustness of the clinical prognostic model of oxidative stress-related gene signatures (GSE31210 and GSE50081). The validation cohort produced results that were similar to those shown in the training set. A poor prognosis was noted in the high-RS group, and a good prognosis was noted in the low-RS group (Figures 7(d)–7(g)).

### 3.8. Expression of RS in Different Clinicopathological Features and Different Molecular Subtypes

To test the link of RS scores with clinical properties of lung adenocarcinoma, the variations of RS scores in various TNM grades, clinical stages, age, genders, status, and clusters were assessed in TCGA-LUAD dataset. The outcomes highlighted that the samples with later clinical stages had higher RS. The RS of male patients was higher in comparison with that of female patients, and the mortality rate of patients with high RS was also higher (Figure 8(a)). Moreover, there were major variations in RS of the three subtypes. The C1 subtype had a higher RS, and the C3 subtype had a lower RS (Figure 8(a)). A comparison between the clinicopathological variations in RS groups of TCGA-LUAD cohort was performed (Figure 8(b)). The outcomes indicated that the high-RS group accounted for more advanced clinical stages, and the proportion of male patients and dead patients was also larger. Additionally, the link between the RS group and the three molecular subtypes we defined earlier was compared. The outcomes revealed that the proportion of the C1 subtype with the worst prognosis in the high-RS group was considerably more in comparison with that in the low-RS group (Figure 8(b)). Afterward, a comparison was done to see if there were prognostic variations in the high-RS and low-RS groups defined in various clinicopathological trait groups. The findings indicated that our risk groups also had good effects on different clinicopathological trait groups. There were major variations in the prognosis of the high-RS and low-RS groups, which showed the efficacy of our risk groups (Figure 8(c)). In general, patients in the high-RS group who had poor survival were generally associated with a higher clinical stage.

### 3.9. Immunological Characteristics of the RS Group

To analyze the immunological variations between various RS groups, the relative abundance of 22 types of immune cells was measured with the help of CIBERSORT. The outcomes indicated that the estimated proportions of 11 immune cells in low-RS and low-RS groups were substantially varied (Figure 9(a)). Moreover, we utilized ESTIMATE for evaluating the immune cell infiltration. The outcomes highlighted that “ImmuneScore” and “ESTIMATEScore” in the low-RS group were considerably higher in comparison with those in the high-RS group, with higher immune cell infiltration (Figure 9(b)). Additionally, RS was also linked with the infiltration level of the following cells: (1) memory B cells, (2) resting CD4 memory T cells, (3) activated CD4 memory T cells, (4) resting natural killer (NK) cells, (5) M0 macrophages, (6) resting dendritic cells, and (7) resting mast cells (Figure 9(c)). As illustrated in Figure 9(d), using ssGSEA analysis, some pathways involving metabolism and cell cycle were positively linked with the RS of the sample (the correlation was greater than 0.3), including DNA repair, glycolysis, and E2F targets. At the same time, the link between RS and inflammatory activity was also compared. The outcomes highlighted that RS had a major negative link with MHC II, HCK, and LCK but a positive link with IgG, interferon, MHC I, and STAT1 (Figure 9(e)).

### 3.10. Differences in Immunotherapy/Chemotherapy between RS Groups

Through the analysis of the expression of genes linked with immune checkpoints in patients of high-RS and low-RS groups, it was noted that 24 immune checkpoint genes were differentially expressed in the RS group, including ADORA2A, BTLA, and BTNL2 (Figure 10(a)). Immunotherapy's possible therapeutic effects in the high and low-risk score groups were assessed. According to the outcomes, the MDSC, CAF, TAM, M2, exclusion, dysfunction, and TIDE scores were considerably different in the RS group (Figure 10(b)). In MDSC, CAF, exclusion, and TIDE scoring, the high-RS group outperformed the low-RS group; in TAMM2 and dysfunction scoring, the low-RS group outperformed the high-RS group significantly. RS had a substantial positive link with MDSC, CAF, exclusion, and TIDE scoring and a significant negative correlation with TAMM2 and dysfunction score, according to subsequent research (Figure 10(c)). Furthermore, we evaluated the sensitivity of the RS group to traditional chemotherapy drugs Vinorelbine, Paclitaxel, Docetaxel, and Cisplatin, and it was noted that the high-RS group showed a higher sensitivity to these four drugs (Figure 10(d)).

### 3.11. RS in Combination with Clinicopathological Properties of Nomogram to Improve the Prognosis and Survival Prediction

The decision tree was first built using the sex, age, TNM stage pathology data, and RS of patients in TCGA-LUAD queue. RiskType, N stage, and stage in the decision tree revealed that four separate risk groupings, low, mediate, high, and highest, were identified (Figure 11(a)). Furthermore, the overall survival rate differed significantly among the four risk classes (*p* < 0.0001), with the highest-RS group having the worst prognosis (Figure 11(b)). Then, researchers looked at the association between the RS group and the four risk subgroups. The risk groupings low RS and mediate RS were all low-RS patients, whereas high RS and highest RS were both high-RS patients, according to the proportional distribution diagram (Figure 11(c)). Simultaneously, it was observed that there were variations in the distribution of molecular subtypes in various risk subgroups, in which the high-RS and highest-RS risk subgroups were dominated by the molecular subtypes C1 and C2 (Figure 11(d)). Univariate and multivariate Cox regression analyses revealed that RS was an independent risk factor linked with prognosis; the HR was 1.92 and 95% CI was 1.65-2.23 (*p* = 1.36*e* − 17). The T stage and N stage were also greatly linked with prognosis (Figures 11(e) and 11(f)). As a result, a nomogram comprising RS and other clinicopathological variables was created for the prediction of the OS of patients suffering from HCC, with RS contributing the most to the nomogram's survival prediction (Figure 11(g)). The anticipated calibration curve of the three calibration points in 1, 3, and 5 years was near the standard curve (Figure 11(h)), indicating the nomograms' effective prediction ability. Moreover, the model's reliability was assessed using the decision curve analysis (DCA). It was discovered that the advantages of RS and nomogram were much greater than the benefits of the extreme curve. In comparison with other clinical-pathological properties, nomogram and RS revealed the strongest ability for survival prediction (Figures 11(i) and 11(j)).

Here, we compare our model with three risk models selected from previous studies: 8-gene signature [23], 13-gene signature [24], and 9-gene signature [25]. In order to make the model comparable to some extent, we calculated the RiskScore of samples according to the corresponding genes in the three models using the same method and conducted a *z*-score for the RiskScore. After the *z*-score, the samples were divided into the high-risk group and low-risk group. The prognostic difference between the two groups was calculated, but the AUC of the 3 models was lower than that of our model (Figure S3A-C). The KM survival curve showed that patients in the low group had better survival of the 3 models (Figure S3D-F). Our model achieves this standard with a relatively small number of genes, giving it a high advantage. In addition, we use C-index (Concordance Index) to evaluate the prediction ability of the model. The C-index of our model is higher than that of the other three risk models (Figure S3G).

## 4. Discussion

As a result of LUAD heterogeneity and the complexity of the tumor microenvironment, in clinical practice, the long-term efficacy of LUAD treatment is still a major problem. It is very important to categorize and refine the appropriate treatment intervention decisions. Several transcriptome-based classifications are widely accepted in LUAD. Yu et al. determined the molecular subtype of LUAD according to genes linked with tumor invasion and constructed a five-gene prognostic grading system [26]. Ma et al. developed the diagnostic scoring model and prognosis model of LUAD according to the m6A regulator. Zhou et al. made a prognosis model according to the gene properties of 9 immune checkpoints to provide the basis for diagnosis, prognosis, and clinical treatment of LUAD [27]. As oxidative stress regulation could not be ignored, we showed the molecular subtype of LUAD from the perspective of oxidative stress.

In this research, 436 genes linked with oxidative stress were chosen from the MSigDB, and 102 genes that were linked with lung adenocarcinoma prognosis were chosen by univariate Cox regression analysis on LUAD samples in TCGA-LUAD dataset. As per the consistent clustering of gene expression profiles of 102 oxidative stress-related genes with substantial prognosis, LUAD patients were categorized into three subtypes. Prognostic analysis indicated that there were major prognostic variations among the three groups, a better prognosis was observed in C3, and a worse prognosis was noted in C1. Moreover, after analyzing the clinicopathological properties, it was noted that in various subtypes, the C1 subtype had an advanced clinical stage and a higher death rate, which was similar to the poor prognosis of the C1 subtype. In TCGA cohort, we discussed the variations of genetic changes in these three molecular subtypes. The outcomes revealed that subtype C1 showed higher fraction altered, homologous recombination defects, arbitrary score, and number of segments and tumor mutation burden. ROS is well known for its ability to produce a variety of DNA damage [28]. Continuous DNA damage is induced by the generation of ROS and the inflammatory cascade, which causes genomic modifications and raises the likelihood of epigenetic changes. The accumulation of epigenetic alterations may disrupt genome-wide cellular signaling systems, promoting malignant transformation and the development of cancer [29].

The sensitivity of several molecular subgroups in TCGA cohort to immunotherapy and traditional chemotherapy medications was also investigated. C3 subtype's TIDE score in TCGA cohort was lower than that of the other two subtypes, indicating that the C3 subtype was more likely to benefit from immunotherapy, whereas the C1 subtype was more susceptible to Docetaxel, Vinorelbine, and Cisplatin. The induction of oxidative stress may result in cancer cells being targeted for death. For effective cancer treatment, a variety of medicines with direct or indirect effects on ROS have been employed [30]. Clinical tumor therapy (radiotherapy, chemotherapy) should take into account the various stages of tumor incidence and progression, as well as innovative antioxidation modulation techniques, in order to improve tumor cell killing while reducing damage to normal cells. Purple shirt medications like Docetaxel can stimulate cytochrome C release from mitochondria and interfere with the electron transport chain, causing the formation of superoxide free radicals and cell death [31]. Oxidative stress is induced by Vinorelbine by consuming intracellular glutathione, and oxidative stress is important in Vinorelbine-induced cell damage [32]. Platinum compounds can potentially cause apoptosis, resulting in high amounts of ROS [33]. It was discovered that endocellular ROS increased obviously under the stimulation of TGF-*β* [34]. As a second messenger in cells, ROS is associated with the EMT process and regulate many signaling pathways in cells, such as the ROS/NF-*κ*B signal pathway [35]. Furthermore, significant discrepancies in activation pathways were discovered between distinct molecular subtypes. Pathways associated with the cell cycle were considerably enriched in the C1 subtype, while EMT-related pathways were significantly enriched in the C2 subtype. As a result, we hypothesized that oxidative stress-related genes used for molecular typing would be important in the immune and tumor microenvironment.

Subsequently, a total of 337 genes were discovered in the three subtypes, and the prognostic risk model was developed by 7 genes (MELTF, PTPRH, LOXL2, RHOV, CPS1, IRX5, and MS4A1) provided by Lasso regression and AIC algorithm. MELTF, also known as MTF (melanin transferrin) or MTF1 (metal-regulated transcription factor 1), as a homolog of iron-binding transferrin, is highly expressed in melanoma, and its expression in normal tissues is low. According to some studies, it can stimulate the migration, invasion, proliferation, and epithelial-mesenchymal transition (EMT) progress of cancer cells and serves as an attractive target [36, 37]. PTPRH, also called gastric cancer-related PTP-1 (SAP-1), together with PTPRB (also called VE-PTP), PTPRJ (also called DEP-1), and PTPRO, belongs to R3 subtype receptor PTP [38]. Sato et al. discovered that PTPRH was regulated epigenetically by DNA hypomethylation and had prognostic importance related to lung adenocarcinoma [39]. Lysyl oxidase like 2 (LOXL2) is a copper- and lysine tyrosyl quinone- (LTQ-) dependent amine oxidase, and it is a part of the lysyl oxidase (LOX) family. Catalyzing the cross-linking of extracellular elastin and collagen is its usual function. It is observed in many reports that the abnormal expression of LOXL2 in different types of malignancies is linked with EMT, metastasis, chemoradiotherapy resistance, worse prognosis, and progression of a tumor [40–42]. Based on the study by Zhang et al., the RAS homologous family member V (RHOV) is majorly involved in LUAD metastasis and may provide biomarkers for prognosis prediction and LUAD treatment [43]. Other research has found that overexpression of RhoV in lung adenocarcinoma promotes lung adenocarcinoma occurrence and progression, as well as EGFR-TKI resistance [44]. CPS1 (carbamoyl phosphate synthase 1) is a rate-limiting enzyme in the first step of the urea cycle and is also required for human liver metabolism [45]. Pham-Danis et al. discovered that inhibiting CPS1 could lower the growth of EGFR mutant non-small-cell lung cancer (NSCLC) cells and stop them from progressing through the cell cycle [46]. A gene encoding CD20 on the surface of B cells called MS4A1 has a major involvement in different pathological environments. Some studies have discovered that MS4A1 is a brain metastasis immune-related gene in LUAD [47]. In embryonic as well as adult development, the IRX5 is a key transcription factor [48]. It has not been reported in lung adenocarcinoma, and detailed studies on it are required.

Finally, the decision tree was built based on the gender, age, TNM stage pathological data, and RS of patients in TCGA-LUAD cohort. The outcomes revealed that only RiskType, N stage, and T stage were left in the decision tree. The nomogram was further created as per the major clinical properties in the univariate and multivariate regression analyses. The analysis of the calibration curve and decision curve highlighted that the model had high prediction accuracy and survival prediction ability. Secondly, selecting genes linked with oxidative stress as target genes was important for the occurrence, development, diagnosis, and treatment of LUAD, and the basis for personalized treatment of patients with LUAD could be obtained using our nomogram model based on TMN staging.

## 5. Conclusions

A new prognostic risk model based on seven genes linked to oxidative stress was developed, and it was found to be effective in prognosis prediction in LUAD patients. The complex molecular function was observed in these 7 genes, with IRX5 being the only one not previously linked to LUAD, which needs to be investigated further. Furthermore, our research highlighted the link between oxidative stress-related genes and LUAD prognosis. Our findings could lead to more precise and tailored treatment for lung cancer patients in clinical trials.

## Figures and Tables

**Figure 1:** Three molecular subtypes of genes are linked with oxidative stress in lung adenocarcinoma. (a) TCGA-LUAD queue sample CDF curve. (b) The CDF delta area curve of TCGA-LUAD queue samples represents the change of the area of each class number *K* under the CDF curve relative to *k* − 1. The abscissa is for the category number *k*, and the ordinate is for the relative change of the area under the CDF curve. (c) Sample clustering heat map when consumption *k* = 3. (d) Prognostic survival curves of 3 molecular subtypes. (e) Heat map of genes linked with oxidative stress having a substantial prognosis in various subtypes of TCGA-LUAD. (f) Distribution of different molecular subtypes in “oxidative stress ssGSEA scores” in TCGA-LUAD cohort. ns: no significance. ^∗^*p* < 0.05, ^∗∗^*p* < 0.01, ^∗∗∗^*p* < 0.001, and ^∗∗∗∗^*p* < 0.0001.

**Figure 2:** The link between the three subtypes and clinical properties in TCGA-LUAD cohort. (a) Distribution of T stage samples in three subtypes. (b) Distribution of N stage samples in three subtypes. (c) Distribution of M stage samples in three subtypes. (d) Stage sample distribution of three subtypes. (e) Age sample distribution of three subtypes. (f) The distribution of sex samples of three subtypes. (g) The status distribution of three subtypes. ns: no significance. ^∗^*p* < 0.05, ^∗∗^*p* < 0.01, ^∗∗∗^*p* < 0.001, and ^∗∗∗∗^*p* < 0.0001.

**Figure 3:** Relationship of the three subtypes with genomic changes in TCGA-LUAD cohort. (a) Aneuploidy score, homologous recombination defects, fraction altered, number of segments, and tumor mutation burden. (b) The distribution of typical immune molecule subtypes in the three subtypes. (c) The mutation properties of the top 20 most important mutant genes with the greatest frequency of mutations in each subtype. ns: no significance. ^∗^*p* < 0.05, ^∗∗^*p* < 0.01, ^∗∗∗^*p* < 0.001, and ^∗∗∗∗^*p* < 0.0001.

**Figure 4:** Immune-associated traits of each subtype. (a) The abundance of each immune infiltrating cell of the 3 subtypes in TCGA-LUAD cohort. (b) Variations in matrix, immunity, and estimated score among the three subtypes in TCGA-LUAD cohort. (c) Differential expression of different immune checkpoint genes of three subtypes in TCGA-LUAD cohort. (d) The results of TIDE analysis among different subtypes in TCGA-LUAD cohort were different. (e) The box plots of the estimated IC50 for Docetaxel, Vinorelbine, Paclitaxel, and Cisplatin in TCGA-LUAD. ns: no significance. ^∗^*p* < 0.05, ^∗∗^*p* < 0.01, ^∗∗∗^*p* < 0.001, and ^∗∗∗∗^*p* < 0.0001.

**Figure 5:** Pathway features of various subtypes. (a) The results of GSEA of different subtypes in TCGA-LUAD cohort. (b) The scores of seven inflammatory-related gene clusters of various molecular subtypes in TCGA-LUAD cohort were varied. (c) The score variation of different molecular subtypes in the iron death pathway in TCGA-LUAD cohort. (d) The scores of different molecular subtypes in the autophagy pathway were different in TCGA-LUAD cohort. (e) The score difference of different molecular subtypes in an angiogenesis-related gene set in TCGA-LUAD cohort. ns: no significance. ^∗^*p* < 0.05, ^∗∗^*p* < 0.01, ^∗∗∗^*p* < 0.001, and ^∗∗∗∗^*p* < 0.0001.

**Figure 6:** Identification of genes related to oxidative stress: (a) univariate Cox regression analysis was utilized for analyzing the differential genes among different subtypes that had an impact on prognosis; (b) Lasso coefficient distribution of 337 genes with prognostic value; (c) using 5 cross-validation for choosing the best parameters in the model; (d) the coefficient of individual genes in the optimal model.

**Figure 7:** Generation and evaluation of the RiskScore model according to the seven genes related to oxidative stress. (a) The risk map of TCGA-LUAD shows the expression, survival status, and risk value distribution of 7 genes related to oxidative stress in each LUAD patient. (b) ROC curve for significance prediction of 1-, 3-, and 5-year OS RiskScore in TCGA-LUAD cohort. (c) Kaplan-Meier curve for OS of LUAD patients in low-risk and high-risk groups in TCGA-LUAD cohort. (d) The ROC curve was utilized for examining the predictive effect of the prognostic risk model in the GSE31210 cohort at one, three, and five years. (e) Kaplan-Meier survival analysis between low-risk and high-risk patients in the GSE31210 cohort. (f) Time-dependent ROC curve of the prognostic risk model in the GSE50081 cohort. (g) Kaplan-Meier curve of the prognostic risk model for LUAD patients in various risk groups in the GSE50081 cohort. ns: no significance. ^∗^*p* < 0.05, ^∗∗^*p* < 0.01, ^∗∗∗^*p* < 0.001, and ^∗∗∗∗^*p* < 0.0001.

**Figure 8:** Association between RiskScore grouping and clinicopathological features. (a) The violin chart shows the RiskScore distribution in TCGA-LUAD queue according to T stage, N stage, M stage, stage, age, gender, status, and cluster. (b) The clinicopathological features of RiskScore groups in TCGA-LUAD cohort, including T stage, N stage, M stage, stage, age, gender, status, and cluster. (c) KM curve of RiskScore in the high-risk and low-risk groups among different clinicopathological groups in TCGA-LUAD cohort. ns: no significance. ^∗^*p* < 0.05, ^∗∗^*p* < 0.01, ^∗∗∗^*p* < 0.001, and ^∗∗∗∗^*p* < 0.0001.

**Figure 9:** Immunological variations among various RiskScore groups. (a) Estimated percentage of 22 different immune cells in different RiskScore groups in TCGA-LUAD cohort. (b) Differences in the matrix, immune, and ESTIMATE scores in the low- and high-RiskScore groups. (c) Pearson correlation analysis in 22 immune cells and RiskScore. (d) Correlation analysis results between pathways with RiskScore correlation greater than 0.3 and RiskScore. (e) Results of correlation between RiskScore and inflammatory activity. ns: no significance. ^∗^*p* < 0.05, ^∗∗^*p* < 0.01, ^∗∗∗^*p* < 0.001, and ^∗∗∗∗^*p* < 0.0001.

**Figure 10:** The role of prognostic risk models in predicting the benefits of immunization/chemotherapy. (a) Expression of genes linked with immune checkpoints in patients with low and high RiskScore. (b) The difference of TIDE analysis results among different RiskScore groups in TCGA-LUAD queue. (c) Correlation between RiskScore and TIDE analysis results in TCGA-LUAD queue. (d) Differential chemotherapy responses in the low- and high-RiskScore groups per the IC50 accessible through TCGA-LUAD database: Docetaxel, Vinorelbine, Paclitaxel, and Cisplatin. ns: no significance. ^∗^*p* < 0.05, ^∗∗^*p* < 0.01, ^∗∗∗^*p* < 0.001, and ^∗∗∗∗^*p* < 0.0001.

**Figure 11:** Nomogram of the prognostic risk model combined with clinicopathological features. (a) Patients with full-scale annotations comprising RiskScore, age, gender, and TNM Stage were employed for developing a survival decision tree to optimize risk stratification. (b) Major variations of overall survival were noted in the four risk subgroups. (c, d) Comparative analysis in different groups. (e, f) Univariate and multivariate Cox analyses of RiskScore and clinicopathological properties. (g) Nomograph model based on RiskScore and clinical factors. (h) Calibration curve of nomograph in 1, 3, and 5 years. (i) Decision curve of nomograph. (j) Different clinical variables predict the prognosis of AUC. ns: no significance. ^∗^*p* < 0.05, ^∗∗^*p* < 0.01, ^∗∗∗^*p* < 0.001, and ^∗∗∗∗^*p* < 0.0001.

## Data Availability

The datasets analyzed in this study were available in GSE31210 at https://www.ncbi.nlm.nih.gov/geo/query/acc.cgi?acc=GSE31210 and in GSE50081 at https://www.ncbi.nlm.nih.gov/geo/query/acc.cgi?acc=GSE50081.

## Supplementary Materials

Supplementary 1 Table S1: a list of 102 genes related to oxidative stress and the prognosis of lung adenocarcinoma.

Supplementary 2 Figure S1: flow chart of the work.

Supplementary 3 Figure S2: functional enrichment analysis.

Supplementary 4 Figure S3: validation of published models. (A) ROC analysis of the 8-gene signature. (B) ROC analysis of the 13-gene signature. (C) ROC analysis of the 9-gene signature. (D) KM survival analysis of the 8-gene signature. (E) KM survival analysis of the 9-gene signature. (F) KM survival analysis of the 13-gene signature. (G) C-index of three risk models.
